# Relaxant Effects of the Aqueous Extract of *Excoecaria grahamii* (Euphorbiaceae) Leaves on Uterine Horn Contractility in Wistar Rats

**DOI:** 10.1155/2021/6618565

**Published:** 2021-04-09

**Authors:** Prosper A. Dabiré, Youssoufou Ouédraogo, Abel A. Somé, Stanislas Sawadogo, Issaka Ouédraogo, Edith M. Ilboudo, Raymond G. Belemtougri

**Affiliations:** ^1^Department of Life and Earth Sciences, Institute of Sciences, 01 BP 1757 Ouagadougou 01, Burkina Faso; ^2^Laboratory of Animal Physiology, Department of Animal Biology and Physiology, University Joseph Ki-Zerbo, 03 BP 7021 Ouagadougou 03, Burkina Faso; ^3^Laboratory of Plant Biology and Ecology, Department of Plant Biology and Physiology, University Joseph Ki-Zerbo, 03 BP 7021 Ouagadougou 03, Burkina Faso; ^4^Laboratory of Entomology, Department of Animal Biology and Physiology, University Joseph Ki-Zerbo, 03 BP 7021 Ouagadougou 03, Burkina Faso

## Abstract

In uterine smooth muscle, the effects of *Excoecaria grahamii* are not yet documented. To fill this gap, we investigated the pharmacological effect of *Excoecaria grahamii* on the contraction of the rat isolated uterine horns. The isolated segments were exposed to different concentrations of the aqueous extract of *Excoecaria grahamii* leaves and pharmacological drugs. The results showed that *Excoecaria grahamii* aqueous extract decreased the amplitude and frequency by concentration-related manner. IC_50_ values were 2.4 and 2.6, respectively, for amplitude and frequency. Our study revealed that the extract did not act through histamine H_2_-receptors or the nitric oxide pathway. It also inhibited uterine contractions induced by oxytocin and potassium chloride (KCl). These data suggest that *Excoecaria grahamii* active compound can be used for calming uterine contractions. The action of *Excoecaria grahamii* showed that it can be useful to fight against diseases which caused uterotonic effects. It can be useful to prevent preterm birth and pains caused by menstruations but further investigation is needed to clarify the mechanism action.

## 1. Introduction

*Excoecaria grahamii*, formerly called *Sapium grahamii*, is a plant used in traditional medicine of Burkina Faso. This plant is known for many therapeutic properties. Indeed, ethnobotanical surveys have revealed that the decoction of the whole plant is used to treat skin diseases [1]. The plant is generally indicated for the treatment of leprosy, ascites, and conditions where the use of a powerful purgative seems necessary; it is also used in the treatment of dysentery and Guinea worm [1]. In the locality of Kombissiri (Burkina Faso), it is used as an insecticide to protect crops [2].

Furthermore, we have notice that *Excoecaria grahamii* is traditionally used to induce abortions [1, 2]. However, studies have not been conducted to examine the abortion activity of *Excoecaria grahamii*. Thus, it can be hypothesized that the aqueous extract of *Excoecaria grahamii* leaves causes an increase on uterine contractions because an increase of uterine contractions during pregnancy is a major risk of abortion.

Scientific investigations on the toxicity have shown that *Excoecaria grahamii* leaves are slightly toxic [3–5]. Other investigations have shown many possible pharmacological properties. In the literature, we found that the aqueous leaf extracts are known to act on the intestinal smooth muscles [2]. This author showed that the aqueous extract and the aqueous extract heated to more than 100°C exerted hypotonifying and hypertonifying effects, respectively. In addition, Belemtougri et al. [6] demonstrated the hypertensive activity of the hydroalcoholic leaf extract while the aqueous extract showed a hypotensive and antihypertensive effect [5]. Chemical analyses of extracts from *Excoecaria grahamii* yielded constituents as anthocyanosides, tannins, saponosides, reducing compounds, oses and polyoses, flavonoids, and triterpene steroids [7].

We noted that all these studies done previously focused on intestinal or vascular smooth muscles. However, the effect of *Excoecaria grahamii* on the rat uterus is not yet documented.

Therefore, this study is aimed at assessing the effect of the aqueous extract of *Excoecaria grahamii* leaves on the contractility of the isolated uterus of nonpregnant Wistar rats and determining its mechanism of action.

## 2. Materials and Methods

### 2.1. Plant Collection and Extract Preparation

The plant sample was collected from its natural habitat in the locality of Kombissiri in the south-eastern region of Burkina Faso, located at 42 km from Ouagadougou the capital of Burkina Faso (11° 55′ 33.8^″^ North; 01°17′10^″^ East). The samples were collected during the dry season and identified by the Herbarium of the Biodiversity Centre of Joseph Ki-Zerbo University, where the voucher specimen (ID No: 16703 and sample No: 6786) was stored. The leaves of the plant were dried in shade at room temperature (30 ± 2°C) for 14 days. The leaves were powdered and macerated using 100 g of powder in one litre (1 L) of distilled water for 24 h. The maceration was done using a magnetic stirrer, and the solution was then filtered using a Whatman No. 2 filter paper and freeze-dried. The powder obtained was yellowish in colour. It was stored at -4°C and used for the different tests. The extraction yield was approximately 13% (w/w).

### 2.2. Animals

Nonpregnant female Wistar rats (200–250 g) were used in this study. The oestrous cycle stages were monitored daily using vaginal smears, and the rats were sacrificed only in the metoestrus or dioestrus [8–12]. Thirty (30) nonpregnant rats were fed with granules containing 29% of proteins provided by the western regional office of the “Centre de Promotion de l'Aviculture Villageoise” (CPAVI) of Bobo-Dioulasso (Burkina Faso), and they were kept at 22 ± 2°C, 60 ± 10% humidity. The rats were submitted to a 12-hour light/dark cycle with food and tap water *ad libitum*. All procedures involving animals strictly followed ethical considerations for scientific research in the Joseph Ki-Zerbo University. The agreement number of ethical committee for this study is CEEA-UJKZ_02.

### 2.3. Isolated Tissue Preparation and Tension Measurement

The study was undertaken at University Joseph Ki-Zerbo. The rats were anesthetized with urethane (15%; 1.5 g/kg) by intraperitoneal route after receiving authorization from the university's ethics committee. The isolated uterine horns were rapidly removed and placed in a physiological solution composed of (mM): 154 sodium chloride (NaCl), 5.4 potassium chloride (KCl), 2 calcium chloride (CaCl_2_), 1.2 magnesium sulphate (MgSO_4_), 1.8 potassium dihydrogen phosphate (KH_2_PO_4_), 22 sodium bicarbonate (NaHCO_3_), and 8 glucose, pH adjusted to 7.4. They were freed of the adhering connective tissues and fat. The isolated uteri were segmented into 10 mm long sections. The part of the horn involved in this experiment is equivalent to the 10 mm section described by Chen et al. [10]. The isolated segment was ligated at both ends, and the lower end was attached to a fixed hook. Then, the uterine segment was mounted vertically in a tissue organ bath containing 10 mL of the physiological solution (pH 7.4 and temperature 37°C) and connected to a force transducer (Model FT03, Grass Instruments, Quincy, MA, USA) using silk threads. The maximum volume of the organ bath was 20 mL. Electrical signals from the transducer were amplified using a ETH-400 bridge amplifier (CB Sciences, Dover, NH, USA) and converted to digital signals to be recorded by a MacLab/8e digitizer (AD Instruments, Castle Hill, NSW, Australia) using the Chart software (v 4.2 for windows, AD Instruments Pty Ltd, Australia). The resting tension applied to the uterine segments was 0.5 g. An equilibrium period of 45 minutes was required to allow spontaneous and homogeneous contractions of the uterus before testing the leaf extract or any other drug.

### 2.4. Drug Challenges

After the equilibrium period, the extract was added cumulatively in the single organ bath containing the physiological solution to successively obtain concentrations of 1, 2, 3, 4, and 5 mg/mL each five minutes of time interval. This allowed measurement of the amplitudes and frequencies of the extract effects.

To determine the inhibitory effect of the extract on H_2_ histamine receptors, the uterine segments were allowed to react with ranitidine (10^−2^ mg/mL) an H_2_-receptor antagonist, for 20 min. Subsequently, the extract was added cumulatively to obtain 1-8 mg/mL in the organ bath. This effect was compared to that of a control carried out with histamine.

In order to investigate a probable interaction of the extract with other mechanisms, substances such as KCl (60 mM, bath concentration), oxytocin (10 mIU/mL, bath concentration), and N^*ω*^-nitro-L-arginine methyl ester (100 *μ*M bath concentration, inhibitor of nitric oxide synthase) were used. These substances were allowed to react with the uterine horn segments for 20 min and used as control. The extract was then added cumulatively to obtain 1–8 mg/mL bath concentrations, as mentioned previously.

### 2.5. Standard Drugs Used for the Experiment

Ranitidine (GlaxoSmithKline laboratory, France) was used as an antihistamine to highlight the possible effect of the extract on histamine receptors.

Histamine (Sigma-Aldrich, UK) was used to induce relaxant effects on rat uterine horns by acting on H_2_-receptors.

N^*ω*^-nitro-L-arginine methyl ester or L-NAME (Sigma-Aldrich, UK), an inhibitor of nitric oxide synthase, was used to highlight the possible effects of the extract on the relaxation mechanism through the nitric oxide pathway.

Oxytocin was purchased from Ciron Drugs (India). It was used to increase uterus contractions and demonstrate the possible inhibition of extracellular calcium by the extract.

### 2.6. Statistical Analysis

The data were analysed with the Graph Pad Prism 5.00 software. The contractile activity of the last 5 minutes in the control solution or positive control solutions (ranitidine, oxytocin, KCl, or L-NAME) was calculated and considered to be 100%. The inhibitory effect of each substance was then calculated by taking into account the control, and the data were represented as a concentration-response curves. The amplitudes and frequencies were the parameters used in the analyses of the observed effects. IC_50_ values were determined, and Student's *t-*tests were used for comparisons. The differences in data sets were considered significant (^∗^) and highly significant (^∗∗^) if the *p* value was <0.05 and <0.01, respectively.

## 3. Results

### 3.1. Effects of the Aqueous Extract of *Excoecaria grahamii* Leaves on Spontaneous Uterine Activities

The aqueous extract of *Excoecaria grahamii* leaves inhibited the basic contractions of rat uterine horns in a concentration-dependent manner (Figure 1). The effect was marked by a decrease in the amplitude and frequency of basal uterine contractions. Marked amplitude reduction appears to begin from 3 mg/mL with very little change at all in frequency except at 5 mg/mL. Total relaxation, which corresponded to 100% of amplitudinal decrease, was achieved at 5 mg/mL. The IC_50_ values for amplitude and frequency were found to be 2.4 and 2.6 mg/mL, respectively (Figure 1(b)). This inhibitory effect occurred immediately after addition of the extract to the isolated organ bath, and the effect was maintained throughout the presence of the extract in the organ bath. At 1 mg/mL, the mean percentage decrease level was about 76 ± 7% and 85 ± 2%, respectively, for frequency and amplitude. Moreover, the extract did not change the basal tone compared to the control, and the contractions returned to normal after the organ was rinsed (Figure 1(a)).

### 3.2. Effects of the Aqueous Extract of *Excoecaria grahamii* Leaves on Uterine Contractions in the Presence of Ranitidine

Histamine was found to induce an inhibition of uterine contractions from 100% to 20 ± 6% between 10^−8^ and 10^−3^ mg/mL (Figure 2(a)). When ranitidine (10^−2^ mg/mL) was added to the physiological solution in the organ bath during 20 min before testing histamine, the effect of histamine was inhibited from 100% to 92 ± 3% (Figure 2(b)). At higher concentrations of histamine (≥10^−4^ mg/mL), the inhibition curve (ranitidine+histamine) was significantly different (*p* < 0.05) when compared to the control curve of histamine alone (Figure 2(c)).

When ranitidine was added to the physiological solution in the organ bath during 20 min before adding the extract, a relaxation was observed and the effects of the extract persisted (Figure 2(d)). The relaxation induced by the extract in the presence of ranitidine was similar to that of the extract without ranitidine. The mean percentage of relaxation was 100% at 5 mg/mL (Figure 2(e)). IC_50_ values were 2.38 and 2.21 for AEEG and ranitidine+AEEG curves, respectively. The effect of the extract in the presence of ranitidine (ranitidine+AEEG) was not significantly different compared to that of the extract alone (AEEG) (p > 0.05).

### 3.3. Effect of the Aqueous Extract of *Excoecaria grahamii* on Uterine Contraction Induced by Oxytocin

Oxytocin, which is clinically used to induce labour, stimulated the basic uterine contractions. It caused an increase in the amplitude, frequency, and basic tone of the uterine horns (Figure 3(a)). In the presence of the aqueous extract of *Excoecaria grahamii* leaves added 5 minutes after oxytocin (10 mUI/mL), amplitude and frequency were decreased (Figure 3(b)). The mean percentages of decreases of frequency are approximately 85 ± 4, 67 ± 6, 37 ± 10, and 19 ± 8% for extract concentrations corresponding to 1, 2, 3, and 4 mg/mL, respectively. About the amplitudes, these decreases were 82 ± 5, 68 ± 15, 57 ± 13, and 29 ± 8%, respectively, for the same concentrations of extract. A complete decrease of mean percentage was observed at the maximum concentration used for this test (Figure 3(c)). The IC_50_ values were 2.86 and 3.78 mg/mL, respectively, for frequency and amplitude.

### 3.4. Effect of the Aqueous Extract of *Excoecaria grahamii* Leaves on KCl-Induced Contraction

KCl (60 mM) induced contraction in rat uterine horns (Figure 4(a)). The addition of the extract decreased the amplitude of the contraction in a concentration-dependent manner (Figures 4(b) and 4(c)). The mean percentage of decrease obtained at 8 mg/mL was approximately 20 ± 3% compared to the control considered as 100% (Figure 4(c)).

### 3.5. Effect of the Aqueous Extract of *Excoecaria grahamii* on Uterine Contractions in the Presence of L-NAME

In the presence of L-NAME, the addition of the extract to the physiological solution led to a decrease in the amplitude and frequency of the contractions (Figure 5(a)). The amplitudes decreased immediately, while a slight increase in the frequency was observed initially from 1 mg/ml to 3 mg/mL, and a subsequent decrease occurred from 3 to 5 mg/mL (Figure 5(b)). The maximum relaxation of 100% was observed at 5 mg/mL concentration.

## 4. Discussion

The results of the present study indicate that aqueous extract of *Excoecaria grahamii* relaxed the rat isolated uterine smooth muscle in a concentration-related manner. Our data have shown that the addition of the extract in the organ bath caused a decrease in the amplitude and frequency of contractions. The myometrial layer of the uterus composed of smooth muscle fibers is known to be primarily responsible for contraction of the uterus [11]. In the nonpregnant uterus, contraction serves to evacuate the sloughed endometrial layer, which occurs in the follicular phase. In some females, this may cause mild to severe pain known clinically as dysmenorrhea [12]. In this work, both amplitude and frequency inhibitions are similar to that of *Omphalocarpum procerum* [13] and *Montanoa tomentosa* [14]. These results are also similar to that of resveratrol, a polyphenol known for inhibiting uterine contractions [15]. Moreover, the previous screening of the plant extracts showed phenolic components such as flavonoids that could be responsible for *Excoecaria grahamii* effects. The effect did not match with the existing literature on the traditional usage of *Excoecaria grahamii* leaf extract, which suggests a probable uterotonic effect [1]. Our study has shown and opposite effect. This opposite effect is probably linked to the difference in receptor composition or distribution between the rat and human uteri.

To understand the mechanism of action of *Excoecaria grahamii*, we investigated on histamine receptors. The results of this study showed that ranitidine could not inhibit the effect of the aqueous extract of *Excoecaria grahamii*, eliminating the hypothesis of the participation of histamine H_2_-receptors. This suggests that the biologically active compounds present in the investigated extract may not be histamine H_2_-receptor agonists [16].

Regarding KCl and oxytocin-induced uterine contractions, the results showed that *Excoecaria grahamii* aqueous extract inhibits uterine contractions induced by KCl (60 mM) and oxytocin (10 mUI/mL). KCl and oxytocin mechanism on uterine contraction involve extracellular calcium influx. So, these substances are used to investigate approximately the potential calcium pathway mechanism of action. KCl activates the L-type calcium channels, leading to a massive influx of calcium ions into the smooth muscle cell of the myometrium [17]. When the calcium level reaches a threshold, this causes a contraction. The KCl-related result shows that the aqueous extract of *Excoecaria grahamii* probably modifies the membrane depolarization or blocks calcium channels.

Likewise, oxytocin acts on specific receptors by activating a G protein. The latter stimulates the release of IP_3_ into the smooth muscle cell of myometrium. IP_3_ blocks the potassium channel SLO 2.1 and gives rise to a membrane current [15]. The latter stimulates the voltage-dependent calcium channels by increasing the influx of calcium through the L-type calcium channels. IP_3_ also stimulates the calcium channel of the sarcoplasmic reticulum (SR), leading to the release of calcium. Calcium release from SR and calcium influx leads to contraction of the uterine smooth muscle [18, 19]. Additionally, the results related to this mechanism of oxytocin-induced uterine contractions suggest that the extract active compound could be an oxytocin antagonist. Our data on the inhibition effects on KCl and oxytocin-induced contractions suggests that the extract could prevent the increase of intracellular calcium in the rat uterine myocytes.

The results showed that L-NAME did not prevent the inhibition of the aqueous extract of *Excoecaria grahamii* on the contractility of the isolated uterus. This effect is similar to that observed by Munglue et al. [20] on *Citrullus lanatus* extract. L-NAME is an inhibitor of NO synthase. The release of NO in the uterus of nonpregnant rats and its effect on uterus regulation have been demonstrated [21–24]. The results of this study indicate that the aqueous extract of *Excoecaria grahamii* cannot act via the nitric oxide (NO) pathway.

## 5. Conclusion

This work is aimed at determining the effects of the aqueous extract of *Excoecaria grahamii* leaves and investigating its probable mechanism of action. Data from the studies have shown that the aqueous extract of *Excoecaria grahamii* has a relaxant effect on rat uterine smooth muscle. The extract active compound is not like histamine H_2_-receptor agonist, and the extract relaxant effect is not via the nitric oxide pathway. The aqueous extract of *Excoecaria grahamii* acts by modifying the contractions produced by oxytocin and KCl. Our results suggest that the active compound of *Excoecaria grahamii* could be important to reduce uterine contractions but further investigation is needed to deepen the mechanism action.

## Figures and Tables

**Figure 1:** Effect of the aqueous extract of *Excoecaria grahamii* on uterine spontaneous contractions. (a) Typical recording; (b) summary for the data (*n* = 6 is the number of rats used).

**Figure 2:** Effect of the aqueous extract of *Excoecaria grahamii* (AEEG) on uterine contractions in the presence of ranitidine. (a) Typical recording showing the effect of histamine on uterine contractions, (b) typical recording of histamine in the presence of ranitidine, (d) typical recording showing the effect of AEEG on uterine contractions in the presence of ranitidine, and (c, e) summaries for the data (*n* = 6).

**Figure 3:** Effect of the aqueous extract of *Excoecaria grahamii* (AEEG) on uterine horns segments precontracted by oxytocin. (a) Typical recordings of oxytocin effect on uterine contractions; (b) typical recording showing the effect of AEEG on oxytocin-induced contractions; (c) summaries for the data (OXT: oxytocin; *n* = 6).

**Figure 4:** Effect of the aqueous extract of *Excoecaria grahamii* (AEEG) on KCl-induced contraction. (a) Typical tracing showing the contraction effect of KCl-induced contractions; (b) typical tracing showing the relaxant effect of AEEG on KCl-induced contraction; (c) recapitulative data, *n* = 6.

**Figure 5:** Effect of the aqueous extract of *Excoecaria grahamii* (AEEG) on rat uterine contractions in the presence of L-NAME: (a) typical recording; (b) summaries for the data; *n* = 6.

## Data Availability

To access the data of this finding, please contact Dr. Dabiré Anankpètinan Prosper at the following email address: prosper.dabire@yahoo.frprosper.dabire@ids-ouaga.bf, Institute of Science, Ouagadougou, Burkina Faso.

## References

[1] Nacoulma O. G. (1996). *Medicinal plants and traditional medicinal practices in burkina faso: case of the central plateau*.

[2] Ouédraogo O. C. (1976). Effet des extraits de feuilles et de racine du *Sapium grahamii* (Stapf) Pax. sur les contractions spontanées du duodenum de lapin et l’iléon de cobaye. *Cames*.

[3] Youssoufou O., Raymond G. B., Dabiré A. P., Belemtougri R. G., Dabiré A. P. (2015). Muscarinic activity of aqueous leaves extract of *Excoecaria grahamii* Stapf 1913 on rabbit blood pressure and toad isolated perfused heart. *African Journal of Pharmacy and Pharmacology*.

[4] Traoré A., Ouedraogo S., Kabore A., Tamboura H. H. (2014). The acute toxicity in mice and the in vitro anthelminthic effects on *Haemonchus contortus* of the extracts from three plants (*Cassia sieberiana*, *Guiera senegalensis* and *Sapium grahamii*) used in traditional medicine in Burkina Faso. *Annals of Biological Research*.

[5] Dabiré A. P., Ouedraogo Y., Belemtougri G. R., Tiendrébéogo M. (2017). Phytochemical and toxicity study of *Excoecaria grahamii* Stapf aqueous extract on female mice. *International Journal of Pharmaceutical Sciences and Research*.

[6] Belemtougri G. R., Samate D. A., Millogo-Rasolodimby J. (1995). *Sapium grahamii* (Stapf) Prain : plante cardiotonique. *Journal of Medicine and Pharmacy*.

[7] Traoré A., Ouedraogo S., Belemlilga M. B., Kabore A., Guissou I. P. (2017). Phytochemical analysis and ovicidal activity of *Cassia sieberiana*, *Guiera senegalensis* and *Excoecaria grahamii* extracts. *African Journal of Pharmacy and Pharmacology*.

[8] Caligioni C. S. (2009). Assessing reproductive status/stages in mice. *Current Protocols in Neuroscience*.

[9] Wray S., Noble K. (2008). Sex hormones and excitation – contraction coupling in the uterus : the effects of oestrous and hormones. *Journal of Neuroendocrinology*.

[10] Chen X., Meroueh M., Mazur G. (2018). Phenylephrine, a common cold remedy active ingredient, suppresses uterine contractions through cAMP signalling. *Scientific Reports*.

[11] Wray S., Arrowsmith A. (2012). *Uterine smooth muscle in: muscle*.

[12] Bulletti C., de Ziegler D., De Polli V., Diotallevi L., Ferro E. D., Flamigni C. (2000). Uterine contractility during the menstrual cycle. *Human Reproduction*.

[13] Bafor E., Eyegbagharen T., Ochoyama E., Idu M. (2020). Ex-vivo inhibition of uterine contractility by the stem bark extracts of *Omphalocarpum procerum* P. Beauv . (Sapotaceae) in mouse models. *Journal of Pharmacy & Pharmacognosy Research*.

[14] Perusquía M., Sánchez E., Ponce-Monter H. (1985). The Zoapatle XI. Effects elicited by Mmontanoatomentosa and Montanoafrutescens on rat uterine strips. *Contraception*.

[15] Hsia S., Wang K., Wang P. S. (2011). Effects of resveratrol, a grape polyphenol, on uterine contraction and Ca2+Mobilization in Ratsin *Vivoandin vitro*. *Endocrinology*.

[16] Bertaccini G., Molina E., Vitali T., Zappia L. (1979). Action of histamine receptor agonists and antagonists on the rat uterus. *British Journal of Pharmacology*.

[17] Amaechina F. C., Bafor E. E. (2016). *In vitro* inhibitory effect of methanol leaf extract of *Stachytarpheta jamaicensis* (Verbenaceae) on non-pregnant rat uterus. *Tropical Journal of Pharmaceutical Research*.

[18] Ferreira J. J., Butler A., Stewart R. (2019). Oxytocin can regulate myometrial smooth muscle excitability by inhibiting the Na^+^-activated K^+^ channel, Slo2.1. *The Journal of Physiology*.

[19] Arrowsmith S. (2020). Oxytocin and vasopressin signalling and myometrial contraction. *Physiology*.

[20] Munglue P., Eumkep G., Wray S., Kupittayanant S. (2013). The effects of watermelon (*Citrullus lanatus*) extracts and L-citrulline on rat uterine contractility. *Reproductive Sciences*.

[21] Jain V., Saade G. R., Garfield R. E. (2000). Structure and function of the myometrium. *Advances in Organ Biology*.

[22] Gangula P. R. R., Dong Y., Yallampalli C. (1997). Rat myometrial smooth muscle cells express endothelial nitric oxide synthase. *Human Reproduction*.

[23] Rosselli M., Keller P. J., Dubey R. K. (1998). Role of nitric oxide in the biology, physiology and pathophysiology of reproduction. *Human Reproduction*.

[24] Shmygol A., Gullam J., Blanks A., Thornton S. (2006). Multiple mechanisms involved in oxytocin-induced modulation of myometrial contractility. *Acta Pharmacologica Sinica*.

